# A Liver Damage Prediction Using Partial Differential Segmentation with Improved Convolutional Neural Network

**DOI:** 10.1155/2022/4055491

**Published:** 2022-02-27

**Authors:** B. Sumathy, Pankaj Dadheech, Monika Jain, Ankur Saxena, S. Hemalatha, Wenqi Liu, Stephen Jeswinde Nuagah

**Affiliations:** ^1^Department of Instrumentation and Control Engineering, Sri Sairam Engineering College, Chennai, India; ^2^Department of Computer Science & Engineering, Swami Keshvanand Institute of Technology, Management & Gramothan, Jaipur, Rajasthan, India; ^3^Department of Electronics & Communication Engineering, ITS Engineering College, Greater Noida, Uttar Pradesh, India; ^4^Indus Institute of Information & Communication Technology, Indus University, Ahmedabad, Gujarat, India; ^5^Department of Computer Science and Engineering, Panimalar Institute of Technology, Chennai, Tamil Nadu, India; ^6^Henan Chuitian Technology Co., LTD, Hebi 458000, China; ^7^Department of Electrical Engineering, Tamale Technical University, Tamale, Ghana

## Abstract

**Background:**

The liver is one of the most significant and most essential organs in the human body. It is divided into two granular lobes, one on the right and one on the left, connected by a bile duct. The liver is essential in the removal of waste products from human food consumption, the creation of bile, the regulation of metabolic activities, the cleaning of the blood by sensitizing digestive management, and the storage of vitamins and minerals. To perform the classification of liver illnesses using computed tomography (CT scans), two critical phases must first be completed: liver segmentation and categorization. The most difficult challenge in categorizing liver disease is distinguishing the liver from the other organs near it. *Methodology*. Liver biopsy is a kind of invasive diagnostic procedure, widely regarded as the gold standard for accurately estimating the severity of liver disease. Noninvasive approaches for examining liver illnesses, such as blood serum markers and medical imaging (ultrasound, magnetic resonance MR, and CT) have also been developed. This approach uses the Partial Differential Technique (PDT) to separate the liver from the other organs and Level Set Methodology (LSM) for separating the cancer location from the surrounding tissue based on the projected pictures used as input. With the help of an Improved Convolutional Classifier, the categorization of different phases may be accomplished.

**Results:**

Several accuracies, sensitivity, and specificity measurements are produced to assess the categorization of LSM using an Improved Convolutional classifier. Approximately, 97.5% of the performance accuracy of the liver categorization is achieved with a 94.5% continuous interval (CI) of [0.6775 1.0000] and an error rate of 2.1%. The suggested method's performance is compared to that of two existing algorithms, and the sensitivity and specificity provide an overall average of 96% and 93%, respectively, with 95% Continuous Interval of [0.7513 1.0000] and [0.7126 1.0000] for sensitivity and specificity, respectively.

## 1. Introduction

Cancer has risen to become one of the most prevalent causes of death in contemporary times, and liver cancer has risen to become one of the three most lethal illnesses in the world throughout time [1]. Oncologists may use segmented liver tumor to confirm changes in tumor size that have occurred. The data may subsequently be used to gauge the patient's reaction to treatment and, if necessary, to offer medical help to the patient. Many applications of a medical image recovery system rely on the classification of medical pictures, which is one of the most important things to consider. When highly varied medical picture data become available, reliable classification algorithms are essential to make appropriate decisions. The CT paradigm is used in clinical diagnostics, which allows radiologists to accurately detect and follow changes in the body's physiological state over time. On CT pictures, distinct tissues in separate lines with varying gray rates may be distinguished, and this information can be used to make a medical diagnosis.

Cancer is the leading cause of death in numerous industrialized countries, particularly in the United States [2]. Cancer diagnosis in general practice is based on scientific and histological information that may be faulty or wrong, leading to inaccurate conclusions. When you look at the human body from the inside out, you will see that the liver is located in the upper abdomen. The liver's purpose is to absorb and eliminate waste from the blood. When there is an excess of waste cells in the liver, a lump of tissue known as a tumor or growth may develop [3]. A tumor may be either benign or malignant. Because benign malignancies are not carcinogenic, they should be removed by surgeons. Likely, benign tumor will not recur after therapy in most cases. A hemangioma is a benign blood vessel mass that has become twisted and crowded. Cancer is a term used to describe tumors that have become malignant. The majority of primary liver tumors arise in the hepatocytes. Hepatocellular carcinoma and malignant hematoma are used to describe this kind of malignancy. In the early identification and treatment of liver cancer, ultrasonography (US), CT, and magnetic resonance imaging (MRI) are the most often used diagnostic imaging techniques. For detecting a wide range of disorders, including colon cancer, CT is the most used and recommended procedure. CT scans allow a surgeon to confirm the presence of a tumor and assess the size, location, and duration of the tumor with pinpoint accuracy [4]. Thyroid cancer radiotherapy, biopsies, and other minimally invasive treatments may be effectively planned and administered after CT scans.

Smoothing is required throughout the file processing process to make extraction and grading more convenient and accurate. As a result, it is essential to have a flawless filtering approach in biomedical image processing. Selecting the most suitable segmentation algorithm for a liver tumor picture is critical for achieving good performance. The unknown component of the liver pictures may be extracted using a segmentation method that is suitable for the situation. The first two steps in the feature extraction process are preprocessing and segmentation, which incorporate feature collecting as a second phase. When a candidate is chosen, the categorization procedure is carried out. Selecting the most appropriate filter for denoising, segmentation, function selection, and a prediction algorithm for categorizing liver tumor pictures is still a significant research challenge to be completed shortly.

Liver tumors, often known as liver cancers or liver growths, are malignancies or growths that develop on or inside the liver [5]. Hêpar is the Greek word for liver, and many different types of tumor may be found in the liver. Depending on the stage of development, this development might be benign (cancerous) or malignant. If the tumour cell is natural, it will be nice to be around. There was something wrong, and as a result, the situation got disorganised, and a glob was formed. This did not turn out well. They turn into cancer cells when their growth and division become irregular and out of control, and the tumor progresses to cancer.

### 1.1. Liver Screening

If a person has cirrhosis or another risk factor, it is essentially crucial to follow medical advice, regardless of whether the individual receives frequent liver cancer screenings or not. Early detection will present a higher possibility of success in treating cancer, that is, if discovered before any symptoms appear. Hepatologists are the doctors who have the most significant expertise in screening primary liver cancer. They are also the most expensive. A biopsy, imaging tests such as ultrasound, CT, or CAT scan, or testing for the chemical Alpha-Fetoprotein (AFP) in the blood, which may be produced by cancer cells, are all options for cancer screening (MRI) [6]. More information about these tests may be found in the diagnostic section of the therapy section of this website. According to the etiology of liver illness, various rules must be followed. Diagnosis is the process of identifying an illness based on its symptoms, indicators, and the after-effects of various analytic procedures. The decision reached as a result of the operation as to whether a tumor is malignant or benign is referred to as a diagnostic outcome. When it comes to diagnosing liver cancer, several tests must be performed, and the doctors may do some preliminary tests to see if the disease has moved to another section of the body from where it originated. This condition is referred to as metastasis [7]. A biopsy is the sole technique for a doctor to determine whether or not a specific region of the body is affected by cancer in most cancer cases. A biopsy is a procedure in which a physician removes a tiny sample of tissue to be tested in a laboratory. A biopsy may not be feasible, in which case the doctor may offer additional tests that may aid in the diagnosing process.

The most prevalent primary liver cancer is hepatocellular carcinoma. Hepatocellular carcinoma (HCC) is more common in persons with persistent liver disorders such as cirrhosis from hepatitis B, or C. HCC is often identified without the need for a biopsy [8].

Physicians consider the following variables when deciding on a diagnostic procedure: The kind of cancer suspected, the signs and symptoms experienced by the patient, the patient's age and medical condition, and the findings of previous medical tests.

HCC may be diagnosed with the use of the tests listed below. It is possible to diagnose each form of cancer with the tests on this list; however, not all tests on this list would be recommended for every individual. Examination of the physical body: If a patient exhibits signs of HCC, the physician will palpate the abdomen to look for lumps, swelling, or other abnormalities in the liver, spleen, or other surrounding organs, among other things. The doctor would also examine for indications of jaundice, which include yellowing of the skin and whites of the eyes and an abnormal build-up of fluid in the abdomen. Tests of the blood: In addition to a physical examination, the physician would most likely do a blood test to check for the presence of a chemical known as AFP [9]. AFP is discovered in high concentrations in the blood of around 50% to 70% of persons with advanced HCC. In addition, the physician would examine the patient's blood to determine whether or not he or she had hepatitis B, or C. Other blood tests may be used to determine how effectively the liver is functioning.

### 1.2. Medical Imaging Techniques

The development of visual representations of regions in the human body is the medical imaging technology used to diagnose medical issues and monitor treatment outcomes. Zia et al. [10] are the most well-known names in the business. The human body is a highly complex system that requires a great deal of attention. In-depth examination of data's static and changing features adds to the accumulation of large amounts of information. One of the most challenging problems for academics and physicians is figuring out how to gather, store, and display massive amounts of information about the body in a way that can be digested, processed, and utilized to develop more helpful diagnostic tools and treatment processes.

In many cases, presenting information in visuals is the most efficient method for solving this difficulty. We, as human beings, are well aware of this efficiency; we have relied on vision more than any other perceived ability to interact with the world around us from our earliest years. Photomicrographs of a dynamic object, such as the human body, capture elements of the entity, such as its transmission, clarity, emissivity, reflectivity, conductivity, and magnetic properties, together with fluctuations in time in each of these attributes. To offer specifics on the fundamental features of the material, images that depict one or more of these characteristics may be analyzed to provide more information. Physicians are increasingly reliant on such pictures to understand the human body better and intervene in the processes of sickness and damage in the patient. Imaging to organize and analyze biological and medical processes is expected to continue to grow in importance, not just in clinical medicine but also in the biomedical research sector that underpins clinical care and its support. A medical imaging method and the process is a technique and process that is used to take pictures of the human body (or parts and functions of the human body) for clinical reasons (medical treatments that are intended to disclose, diagnose, or analyze illness) or medical science research (including the study of normal anatomy and physiology). It is possible to do medical imaging on excised organs and tissues, although this is not often referred to as medical imaging and is instead considered part of pathology rather than medicine. Computer-Aided Diagnosis (CAD) systems categorize medical images as a fundamental approach. In medical imaging, traditional approaches focus primarily on form, color, texture elements, and their combinations. The majority of these features are issue-specific and complementary in previous studies. As a result, the system is unable to construct representations of high-level issue domain ideas and has a weak model generalization capacity, as seen in Figure 1.

Recent deep learning algorithms give an efficient solution to design an end-to-end model that can calculate final classification labels from the raw pixels of medical pictures using just the raw pixels of medical images. On the other hand, deep learning models suffer from high computing costs and constraints in the model layers and channels as a result of the high resolution of the medical pictures and the short dataset size, respectively. A large number of algorithms are being used to tackle these challenges.

*Classification* is a supervised learning strategy used in deep learning and statistics, in which the computer program learns from the input data and then utilizes this learning to categorize fresh observations. There are many applications for classification issues, including voice and handwriting recognition, biometric identification, document categorization, and illness classification, to name a few [11]. More research is required to increase the accuracy, efficiency, and robustness of liver CT segmentation. The use of enhanced edge detection techniques, parallelization, and the combination of diverse approaches may be the most effective means of developing improvements in liver CT segmentation methods. To correctly identify and segment tumor sections from liver CT scans, even when the pictures are noisy, it is necessary to conduct this study and create unique techniques. During the first phase of this project, the enhanced design was implemented. The segmentation of the liver CT image is accomplished using the ANN approach. This approach is more often used for grouping large amounts of data quickly and effectively. This means that image processing methods, particularly segmentation approaches, may benefit from it. Although this approach does not need any training data, it does require initial segmentation settings, which are the primary benefit of this technique.

A new enhanced residual GoogleNet CNN approach [12] is suggested to increase the performance of the classification process. According to the current study's findings, uniformity in lesion segmentation leads to better results in patients. It has been observed that the present techniques make use of the form specification, which lacks certain qualities such as homogeneity. There are 24 approaches for identifying abnormalities in liver CT scans that are comparable to one another but we only take a restricted range of parameters into account. Such strategies do not improve the performance and accuracy of verification operations.

### 1.3. Limitations of Existing Approaches

Compared to other techniques, these do not consider several different categorization functions. The decreased accuracy of the diagnosis and the increased temporal variability made it challenging to detect liver cancers [13]. It is evident from the more rigorously constructed and verified research that machine learning approaches may be utilized to significantly (15–25 percent) enhance the accuracy of predicting cancer susceptibility, recurrence, and death in patients with cancer.

### 1.4. Contribution of the Proposed Work

Following are the aims of the proposed work:

- Develop a unique machine learning soft optimization and deep learning method for liver image classification and segmentation from CT pictures;
- Detect and categorize abnormality in liver CT images; and
- To develop an effective liver tumor detection and classification strategy that considers a more significant number of characteristics.

The research team measured classification accuracy and time complexity to evaluate the liver tumor growth methodologies. Among the achievements made by the current research team is the invention of a filter performance measure for liver image preprocessing.

Biomedical Applications of Intensive Artificial Neural Network (ANN) for Liver Tumor Classification in Health Care [14]

The details of the bulk of the tumor have been improved using the Clinically Visual Deep Neural Network (DNN) technique based on volumetric analysis for liver tumor categorization. The remaining sections of the paper are grouped as follows: The background analysis from the current technique is included in Section 2 of the report.  Section 3 contains the technique for segmenting the liver from other organs and the segmentation of liver cancer from the separated liver pictures.  Section 4 contains the methodology for segmenting the liver from other organs.  Section 3 describes the categorization of the proposed Convolutional Layer, followed by Section 4, which contains the experimental findings and discussion of the proposed Convolutional Layer.  Section 5 concludes with a discussion of future work and provides a conclusion.

## 2. Theoretical Analysis of the Existing Research Methodology

Generally speaking, cancer may be characterized as a condition in which aberrant forms of cells proliferate and spread uncontrollably throughout the body. In medical terminology, the word “neoplasm” (which refers to new growth) should be used rather than the phrase “cancer.” “Benign” neoplasms are those that have just the feature of confined growth and are thus categorized as such. A study by Miller et al. was published in 2019 [15]. *Malignant tumors* are defined as those that have the characteristics of invasiveness and the ability to metastasize in addition to their primary characteristics. The word cancer is typically reserved for certain forms of tumor development. Although the term “tumor” really refers to a “local swelling,” it is often used interchangeably with the term “cancer” and will continue to be used in this manner in the future.

A benign tumor is often surrounded by fibrous tissue, making surgical excision of the whole tumor relatively straightforward. When examined under a microscope, the cells of a benign tumor seem to be very similar to the cells of the surrounding healthy tissue. Compared to normal cells, which often include a high proportion of cells in a growth-arrested or quiescent stage of the cell cycle, benign tumor cells typically contain an increased proportion of cells in the mitotic (dividing) stage of the cell cycle. The opposite is true for advanced malignant tumors, which, although may be encapsulated in the early stages of their growth, do not have well-defined borders and instead have spread into the surrounding healthy tissues. Furthermore, they may be distinguished from normal and benign tumor cells by their appearance. Not only do they spend most of their time in the mitotic stage of the cell cycle, but they also have an abnormally large number of chromosomes (aneuploidy).

Using a robotized framework for the segmentation and classification of liver tumor, Vadali et al. [16] developed an efficient and straightforward approach. Specifically, the suggested framework includes preprocessing, segmentation, post-processing, and the final categorization into a benign and malignant tumor, among other things. The picture is downsized to a resolution of 256 × 256 pixels during the preprocessing step. During the segmentation step, the level set approach is linked to segmenting the suspected region. The area of fascination is identified from the initial photograph when it comes to the post-processing step. Finally, the Pseudo Zenerike minute and the GLDM are used to highlight extraction from a CT picture. These components are provided to contribute to the SVM to determine whether the tumor is benign or malignant. The SVM is prepared to make use of four different photos. The suggested framework has an accuracy rate of 86.7 percent, which is rather impressive. A new framework, the CFCSA, was suggested by Anter and Ali [17], in which the crow search algorithm uses the global optimization strategy to overcome the sensitivity of the local optimization technique.

In this approach, the fuzzy c-means (FCM) objective function is employed as a cost function, and the chaotic crow search optimization algorithm is used to find the optimum solution. Benchmarking is performed against the binary crow search algorithm (BCSA), chaotic ant lion optimization algorithm (CALO), binary ant lion optimization algorithm (BALO), and bat algorithm relevant methodologies to see how well the new algorithm CFCSA performs. In this study, the proposed CFCSA algorithm is compared to other algorithms such as the BCSA, CALO, BALO, and bat algorithms. The algorithms are tested in the following areas: diabetes, heart disease, Radiopaedia CT liver imaging, breast cancer, lung cancer, cardiotocography, ILPD, liver disorders, hepatitis, and arrhythmia. According to Diana et al. (2020) [18], the optimal DNN parameters yield the best optimum performance over the datasets under consideration. Wang et al. [19] proposed an efficient sampling strategy based on Inverse Random Under Sampling (IRUS) to solve the difficulties of class imbalance to improve efficiency.

IRUS undersamples the majority class, resulting in several unique partitions, each of which contains samples from the minority and majority classes separated by a border. An optimization strategy based on the Artificial Plant Optimization (APO) algorithm is also presented to select the most effective and efficient features and parameters of classifiers to increase the effectiveness and efficiency of classification. Using an optimization method, the number of iterations and computation time required for feature selection and parameter selection for classifiers that distinguish between HCC recurrence and nonrecurrence are reduced. Support Vector Machine (SVM) and Random Forest (RF) classifiers categorize patients as having or not having HCC based on optimum characteristics and parameters derived from the data. A review of the principles of deep Improved Convolutional Neural Networks for image classification was published by Qin et al. [20], followed by deep learning to categorize localized hepatic lesions on multiphase CT images of the liver. Nanda et al. [21] investigated deep learning approaches as a first and primary method for extracting the liver from an abdominal CT scan and then, as a result, for segmenting the lesions from a tumor-ridden liver after the liver had been extracted.

To segment lesions, once a tumor has been discovered in the liver by GA-ANN, which has been fed textural liver data using LTEM for its classification method, a cascaded model of Improved Convolutional Neural Networks is utilized. To tackle the segmentation of liver tumor in CT abdominal images, Budak et al. [22] first defined the issue as a classification problem and then solved it using a cascaded classifier architecture based on Deep Improved Convolutional Neural Networks. It was built and taught to detect liver regions and lesions in CT scans with low picture quality using two deep encoder-decoder Improved Convolutional Neural Networks (CNN). In another way, an EDC segments the liver picture and uses the segmentation as input for training a second CNN. Once the tumor areas inside the liver ROI regions have been segmented as anticipated by the first EDC, the second ED CNN may be applied. The segmentation of the hepatic tumor inside the liver ROI also considerably reduces false-positive results.

To quantify the performance of the proposed model, it was tested against a publicly available dataset (3DIRCADb), and many metrics were utilized to assess its performance. Ben-Cohen and colleagues (2018) [23] intended to aid in the identification of liver metastases for CT scans, and it makes use of a completely innovative network (FCN) for both the overall background and local patch detection using a super-pixel sparse classification. The use of CT  scans is emphasized unusually. The importance of finding liver metastases, especially tiny metastases, in the early identification of liver cancer cannot be overstated when it comes to the early detection of liver cancer. Ben-Cohen and colleagues (2016) have examined CT exams for liver segmentation and identification of liver metastases, with the entire revolutionary network (FCN) being the most promising. FCN has shown to be quite effective for semi-segmentation. Hawkins et al. have developed a novel machine learning approach to diagnosing HCC in 165 patients, which is based on machine learning (2019) [24].

Maaitah et al. [25] developed an intelligent model for liver illnesses that was built on the Fuzzy Neural System (FNS) and other techniques (FNS). Fuzzy systems and neural networks (FNS) are being investigated to identify liver problems in this context. The FNS's structure and learning method are both given in detail. Wang et al. [19] suggested pretrained deep CNNs on picture patches focused on medical abnormalities and then merged them with class activation mappings and region proposal networks to develop abnormality detectors for medical abnormalities. They were using deep transfer learning algorithms. The findings are compared with the results of three other standard classifier algorithms to increase the classification accuracy of the method. A Deep Improved Convolutional Neural Network was used to develop a technique for identifying liver tumor candidates from CT scans, which was published in 2017. For liver disease screening, Yao et al. [26] suggested a densely connected deep neural network (Dense DNN), which was trained using the most widely used liver function tests (LFTs) and demographic information of individuals.

The suggested approach includes a mechanism for identifying liver tumor while limiting bleeding, particularly on CT images, and when there are a large number of lesions, which is particularly important [27]. According to the current study's findings, uniformity in lesion segmentation leads to better results in patients. It has been observed that the present techniques make use of the form specification, which lacks certain qualities such as homogeneity. It is possible to develop comparable approaches for identifying abnormalities in liver CT scans that merely consider a limited number of features. Such strategies do not improve the performance and accuracy of verification operations. Compared to other techniques, these do not consider several different categorization functions [28]. The decreased accuracy of the diagnosis and the increased temporal variability made it challenging to detect liver cancers.

## 3. Methodology of Proposed Screening Technique with Various Stages

As a result of the aggressive nature of liver cancer's growth, few treatment choices are available to patients. Many low- and middle-income countries are under tremendous financial strain to provide adequate treatment for people with liver cancer. Having already reliable estimates of liver cancer incidence will assist in concentrating attention on the need to track liver cancer and enable optimal treatment for people diagnosed with the disease [29]. To accurately and timely predict liver cancer, it is necessary to develop suitable prediction methods for the disease.

Figure 2 represents the flowchart of the proposed work. A CT scan is a noninvasive diagnostic imaging technology that uses a mix of X-rays and computer tomography to create horizontal or axial pictures of the liver, which may be used to diagnose liver disease [30]. As a result, image processing–based research contributes to the advancement of liver cancer therapy. In computer tomography, the X-ray beam travels around the body in a circle surrounding the patient. It provides a new perspective on the same organ in this way. CT scans may be performed with or without “Contrast,” which is a sort of substance that is taken orally and put into an intravenous (IV) line to cause the liver or tissues under observation to become more visible on the screen. The liver is the biggest organ in the body, and it is placed behind the right rib cage and below the base of the lung. It is involved in the digestion of food.

Blood cells are filtered, nutrients are processed and stored, and part of these nutrients is converted into energy [31]. It is also responsible for the breakdown of hazardous chemicals. The left and right lobes of the liver are the two primary hepatic lobes. The quadrate and caudate lobes are visible when the liver is examined below the surface, indicating two extra lobes. Hepatocellular carcinoma (HCC) develops when the liver cells grow out of control and spread to other parts of the body. It is the most common kind of cancer in the United States. Primary hepatic cancers can form when the cells exhibit aberrant activity. According to reports, liver cancer is the second most common disease to cause death in men and the sixth most common cancer to cause death in women. In 2008, around 750,000 individuals were diagnosed with liver cancer, with 696,000 people dying due to the disease. Males get infected at a rate that is twice as high as that of females worldwide. Virus-induced hepatitis may result in the development of liver cancer, which is much more severe. It is estimated that over 1.45 million fatalities occur each year as a result of this virus, according to the World Health Organization [32]. According to the World Health Organization, at 7 percent, Egypt was identified as the nation with the highest prevalence of adult hepatitis C (HIV) infection in 2015. The technique presented in this paper was evaluated using datasets made accessible to the public.

First and foremost, the LiTS dataset was used, which contains 131 CT scan pictures and their corresponding ground facts (clinical annotation). It should be noted that the LiTS dataset also contains a collection of 70 CT scans for testing reasons. However, these pictures do not have any associated annotations [33]. As a result, only the 131 annotated CT scans were considered in this study. There are 24 photos accessible in JPEG format, which were all taken from a DICOM file with dimensions of 630630 pixels and a bit depth of 24 bits.

### 3.1. Noise Reduction Using Pre-Processing

The preprocessing stage of the diagnosis of liver cancer is the first step in the procedure. Preprocessing is necessary to guarantee the long-term viability and usage of a database. Any step seems to be critical in image processing workflow to achieve this. Filters and histogram equalization methods are used to preprocess unneeded error identification before the actual error detection takes place. Noises may be eliminated using a CT image available at this stage. In nonlinear optical filtering systems, the Adaptive Median Filter (AMF) is often used to remove noise from images or signals, and it is also known as the adaptive median filter. A noise reduction approach is a standard preprocessing method for increasing efficiency. When a CT scan is taken, preprocessing is done to improve the picture's contrast. Histogram equalization is often used to improve picture consistency by balancing the histograms.

*Histogram Equalization* is a computer-assisted procedure used to improve the contrast of photographs. The most common sensitivity values are significantly improved, i.e., the picture intensity range is significantly widened. It makes it possible to reduce local contrast to improve ties between areas. As a result, after applying the histogram equalization, the average contrast of the photos is enhanced by a significant amount. Equation (1) represents the intensity increment in the input image

Let *q* denote the normalized histogram of each possible intensity. Hence,

(1) $$\begin{array}{c} q^{\underline{x}}=\left(\text{Intensity of}\frac{\text{image}}{\text{total}}\text{number of pixels}\right). \end{array}$$

The histogram equalized image can be defined as

(2) $$\begin{array}{c} Z_{x,y}=\text{base}\left(\left(Z-1\right)\overset{c_{4}}{\underset{y=0}{\sum }}xq^{z}\right), \end{array}$$

where the base is the integer that is closest to the given value. This is the same as converting the pixel intensity but in reverse.

(3) $$\begin{array}{c} \frac{\partial O}{\partial y}\left(\overset{O}{\underset{0}{\int }}yqO\left(y\right)da\right)=\partial O\left(O\right)\left(y^{-1}\right)\left(O\right)\frac{d}{dO}. \end{array}$$

This is where, at long last, the probability distributed uniformity function may be expressed as ∂*O*/∂*y*.

Equations (2) and (3) represent the preprocessing of the input image. While the results show that the equalization procedure utilized produces flat histograms, it may also soften and enhance the appearance of histograms.

### 3.2. Liver Segmentation Using Partial Differential Technique

In recent years, it has become an increasingly critical and time-consuming effort to segment both the liver and the tumor area. This is accomplished by developing multiple segmentation methods that segment the picture using different modalities. The approaches used for segmentation are classified into three categories: manual segmentation, semi-automatic segmentation, and fully automated segmentation. Medical specialists do manual segmentation of images layer by layer. The liver borders are detected by two distinct radiologists or by the same radiologists at various times in a single picture when manual segmentation is performed. The structure and observation of the medical pictures are explained using this sort of a segmentation method. There are many issues in this area, the most significant of which is reducing picture quality and the increase of artifacts. Equation (4) represents the input segmentation from another organ in the image. L be the input pixel, and O be the intensity of the image.

(4) $$\begin{array}{c} L\left[y\right]=O\left[y\right]+S\left[o\right]+\phi ,y\in S, \end{array}$$

subject to the initial conditions

(5) $$\begin{array}{c} v\left(y,0\right)=h_{0}{\left(y\right)}_{+}\;v_{t}\left(y,0\right)=h_{1}\left(y\right),\ldots ,v_{t}^{\left(x-1\right)}\left(y,0\right)=h_{-1}\left(y\right), \end{array}$$

and spatial conditions are represented in

(6) $$\begin{array}{c} u\left(\theta ,t\right)=h_{0}\left(t\right),\;u_{z}\left(0,t\right)=\hbar_{1}\left(t\right), \end{array}$$

where *L* is the *o*^*th* ^ order derivative w.r.t “*t*,” *R*[1] is a linear operator and *NH* is the nonlinear operator with degree three. And, *ϕ*=*ϕ*(*x*, *t*) and *u*=*u*(*x*, *t*) are two types of functions: known and unknown. Manual segmentation has many significant problems, the most significant of which are the huge number of picture slices required, the lengthy time required, and the lack of satisfactory results. Furthermore, the process of creating a separate dataset is a time-consuming and difficult one. A semi-automatic segmentation system has been created in response to these challenges, which interactively determines the seed sites for determining the liver's border. As a result of this method, we first apply the Laplace transformation to equation (7) concerning the variable *t*, and we get

(7) $$\begin{array}{c} v\left(y\right)=L\left[O\left[v\left(y\right)\right]+S\left[v\left(y\right)\right]\right]+L\left[\phi \left(y,x\right)\right]. \end{array}$$

By using I.C. (7), we get

(8) $$\begin{array}{c} t^{o}\tilde{v}\left(y,t\right)=i\left(y,t\right)+L\left[O|v\left(y,x\right)\right]+G\left[v\left(y,x\right)\right]+\tilde{\phi }\left(y,t\right), \end{array}$$

where

(9) $$\begin{array}{c} \overset{⟶}{i}\left(y,t\right)=\overset{1}{\underset{s=0}{\sum }}xt^{\left(s+1\right)}\mu_{m}^{2}, \end{array}$$

and *u*(*y*, *x*) and $\overset{⟶}{\phi }\left(y,x\right)$ are the Laplace transformed forms of *u*(*y*, *x*) and *ϕ*(*y*, *x*), respectively.

Now, dividing by *t*^*o*^ on both sides, we get

(10) $$\begin{array}{c} u\left(x,s\right)=\left[\left[\frac{h\left(x,s\right)}{s^{n}}+\frac{1}{s^{n}}L\left[Nu\left(x,t\right)\right]+R\left[tu\left(x,t\right)\right]\right]\right]+\frac{\tilde{\phi }\left(y,x\right)}{t^{o}}, \end{array}$$

where *x*, *y* represent the pixels rows and columns, respectively, with the intensity level and smoothening range as t

(11) $$\begin{array}{c} \tilde{f}\left(y,t\right)=\frac{i\left(y,t\right)}{t^{o}}+\frac{o\left(x,s\right)}{s^{n}}. \end{array}$$

Now, we apply inverse Laplace transformation on equation (11) concerning  8^7^, and then we get

(12) $$\begin{array}{c} Vx=C^{-1}\left[\tilde{f}\left(x,y\right)\right]+C^{-1}\left[\frac{1}{y^{o}}L\left[Ov\left(y,u\right)\right]+S\left[v\left(y,t\right)\right]\right]. \end{array}$$

In the second step, we apply a differential transformation on equations (11) and (12) concerning  ^4^*x*′, and we get

and

(13) $$\begin{array}{c} V_{0}\left(u\right)=h_{0}\left(u\right),\;U_{1}\left(u\right)=i_{1}\left(u\right), \end{array}$$

where *V*_*u*_(*v*) and *G*_*l*_(*v*) are the differential transforms of *v*(*x*, *y*) and *z*(*x*, *y*), respectively The closed-form of the solution can be expressed as follows using the aforementioned recurrence equation and initial conditions.

Using this method, it is simple to forecast the properties of the picture being created. The segmentation approach in this work is based on gray scales, which are employed in conjunction with a computer. Specifically, the difference in size between big and tiny pixels surrounding the object's edges is assessed.

(14) $$\begin{array}{c} X^{\text{segment}}=\overset{o}{\underset{s}{\sum }}xV_{2}\left(V_{x},V_{y}\right)\cdot Vo\cdot log_{c_{i}}+\gamma \int^{}c_{i}dy, \end{array}$$

where *W*^Segmentation ^ is the watershed segmentation, *V*2 is the velocity gradient, *V*_*x*_, *V*_*y*_. When a pixel value is low or high, the image's spatial size is represented by log (*c*_i_). When a frequency coefficient is represented by a distance between pixels, the image's spatial size is represented by log (*c*_i_).

### 3.3. Liver Cancer Cells Segmentation Using Level Set Methodology

The conclusion of the local segmentation had been improved with the *i*th slice of all *n* slices, for more precision, and with the use of the true benefits of the Force Function (FF) function, which had been implemented. Geodesic Active Contour (GAC), as well as the Chan-Vese (CV) models, is used in this modification. There are values for the SPF function that are in the range [−1,1]. It altered the signs of the pressure forces within and outside the zone of intersection, causing the contour to shrink when the item was outside the intersection region and to grow when the object was inside the intersection region.

In equation (15), the SPF function is created in the following manner

(15) $$\begin{array}{c} fn\left(j\left(y\right)\right)=\frac{v\left(y\right)-d_{1}+d_{2}/2}{n\left(\left(y\right)-d_{1}+d_{2}/2\right)},y\in \Omega , \end{array}$$

open function of *H*^2^, *j*(*x*) is the given image in Ω, *d*_1_ and *d*_2_ are defined in equations (16) and (17), respectively.

(16) $$\begin{array}{c} d_{1}\left(\phi \right)=\frac{\int_{\Omega }\left(y\right)I\left(\phi \right)dy}{\int_{i}I\left(\phi \right)dy}. \end{array}$$

Here, in the Heaviside function, *I*(*ϕ*) is approximated by a smoothed functional *I*_*F*_ which is defined by equation (17).

(17) $$\begin{array}{c} I_{d}\left(A\right)=\frac{1}{2}\left(1+\frac{2}{\pi }\text{arctan}\left(\frac{\pi }{j}\right)\right). \end{array}$$

The significance of equation (17) may be described in the following manner. Even if the intensities within and outside the object are homogeneous and *c* 1*c* 2, it is evident that Min (Jy)d1, d2 Max (J y), and the equal signs cannot be reached simultaneously everywhere contour, which dominates, is present. As a result, we get the following equation:

(18) $$\begin{array}{c} \text{Min}\left(1\left(x\right)<\frac{d_{1}+d_{2}}{2}\text{Max}1\left(y\right)\right),y\in \Omega . \end{array}$$

When the object is in the opposite position, the function is defined by substituting the fn function, in Equation 18 in the level set formulation, we derive as in the following:

(19) $$\begin{array}{c} \frac{\partial \phi }{\partial t}=fn\left(j\left(y\right)\right)\cdot \left(\text{div}\left(\frac{\nabla \phi }{\left[\nabla \phi \right)}+\alpha \right)|\nabla \phi 1+\nabla fnm\left(y\right)\right)\cdot \nabla \phi ,y\in \Omega . \end{array}$$

A gaussian filtering technique is used to further regularize the degree of regularity to prevent the re-initialization procedure. div(/(||))|| is used to represent Gaussian vectors, which makes the term *fn*(*I*(*x*)) in equation (19) superfluous. As a result, the level set formulation may be simplified in equation (20)

(20) $$\begin{array}{c} \frac{\partial \phi }{\partial t}=spf\left(I\left(x\right)\right)\cdot a|\nabla \phi |\text{,}x\in \Omega , \end{array}$$

The finely segmented liver pictures, referred to as slices, are the result of a level set process that ensures correct closeness on both sides of the liver image.

### 3.4. Feature Extraction and Classification of Liver Cancer Cells

Following the segmentation step, the Gray Level Co-occurrence Matrix (GLCM) may be used to pick the characteristics that are of interest. When used in conjunction with the Gray Level Co-occurrence Matrix approach (GLCM), it is possible to derive second-order statistical texture attributes. The approach has been employed in a variety of applications, and the presence of three or more pixels may be noticed in the third and higher-order textures, indicating that the technique is being used.

Figure 3 represents the feature extraction of DVW. Because it is an arithmetical function, the GLCM can effectively eliminate artifacts in most cases. It is also possible to maintain the accuracy of the picture. It is possible to extract the picture for use in the research process. GLCM can determine the frequency of the pixels with a defined level of accuracy. The single-pixel in issue is to be questioned here, and another pixel is to be referred to as the *l* route and the neighboring value detachment of *m*, which are two different pixels. Ordinarily, *m* only acquires a single value and may profit either way. The generated directional value may then be used to eliminate the properties of the pictures that were utilized in the segmentation procedure.

(21) $$\begin{array}{c} Q\left(n,t\right)=H\left(n,t,p,\phi \right)\overset{i}{\underset{n=1}{\sum }}t\overset{i}{\underset{t=1}{\sum }}tH\left(n,t,p,\phi \right). \end{array}$$

G represents the frequency vector, *m* represents the frequency of the particular component that will generally have the pixel values of *n*, and *H*, *p* represent the normalized constant, where *P* represents the features of an image, (*n*, *t*) represents the component of the *n*, and *H*, *p* represent the normalized constant.

Improved Convolutional Neural Network (ICNN) is a neural network that performs the classification and grouping of pictures quickly and efficiently. The raw pixels of cell photos are used to build the highlight representations in this approach, and the pixel is acquired by using a hand-created system as in previous ways. In addition, the characterization layer is mutually advanced with these component descriptions to predict the class for each cell image in the database. The following opinions are included in the present study and broadened: A more detailed and point-by-point representation of the ICNN classifier structure is shown. Various critical components for putting together this structure are discussed and provisionally considered. This paper presents three main findings:

Figure 4 represents the classifier structure. The role of pivoting cell pictures in information growth is dissected from top to bottom. The suitability of cell picture veils for this grouping assignment is examined, and an illustration of the astounding versatility of the ICNN-based characterization framework to various datasets is provided. Furthermore, further exploratory connections between the ICNN-based structure and the cutting-edge hand outlined shallower grouping models are aimed to illustrate the focus points of the ICNN classifier system–based cell picture classification, notwithstanding the above. When it comes to producing tests based on learning references after sparsity has been determined, the ICNN yield, which includes the sparsity level and records of initial coefficients in insufficient vectors, are used as the two arrangements of components for creating the NN. The recommended diminutive size ICNN grouping is applied in this approach, which uses 3D stomach CT scans in a prepared pipeline to natural criminologists. The International Convention on Nuclear Nonproliferation is characterized as follows:

(22) $$\begin{array}{c} NZC=\;\overset{1}{\underset{i}{\sum }}x\left\|y_{i}-D_{xi}\right\|2\leq OjRMSE^{2}. \end{array}$$

For each dictionary set *D*, ND denotes the number of sparsity levels present, NZC the intended sparsity level and an average number of nonzero coefficients, and RMSE the reconstruction of error or root-mean-square error, respectively. It is input into the ICNN classifier, and the weights are changed until the ICNN returns results that are less than 2.0 for benign instances of liver tumor and more than 2.0 for malignant cases of liver tumor, respectively.

## 4. Experimental Analysis of Proposed Work

The proposed work is implemented using MATLAB software with training and testing images. In this step, two photos of malignant liver tumor are taken from the datasets that have been utilized.

CT scanning has risen to become an essential imaging technique in diagnosing liver tumor. Different studies have utilized different methodologies for classifying liver development based on CT.

Figure 5 represents the segmentation outcomes of the proposed work. The accuracy, sensitivity, and specificity of the suggested approach have been examined, as well as its overall performance

Figure 6 represent the proposed liver segmentation techniques. According to relevant features, the number of liver cancers that are accepted in the result when compared to other tumors, whereas specificity (irrelevant features) refers to the number of nonliver tumors that are rejected in the outcome when compared to other tumors.

The overall accuracy is applied to the end performance, whereas the sensitivity is applied to the acceptance capacity.

The equation is given below.

(23) $$\begin{array}{c} \text{Sensitivity}=\frac{\text{TP}}{\text{TP}+\text{FN}}, \end{array}$$

(24) $$\begin{array}{c} \text{Specificity}=\frac{TN}{TN+FP},\\ \text{PPV}=\frac{TP}{TP+FP}. \end{array}$$

- True Negative (TN): When it is (F) the samples can be classified or false (F)
- False Positive (FP): When it is (F) the samples can be cl + assified as (T)
- False Negative (FN): when it is (T) the sampled can be classified as (F)

To evaluate how well a classification system performs, accuracy is the most widely utilized parameter. The degree to which classifying rules square measure accuracy determines a classification system's accuracy.  Table 1 shows the feature value of the images.

The values are shown in parentheses. The categorization is based on the values of these feature attributes. Following that, the outputs of the feature extraction vectors are trained, and the accuracy of the performance using different classifier approaches is compared. As shown in Table 2, the sensitivity, specificity, and accuracy of the different classifiers are tested in terms of the sensitivity, specificity, and accuracy using a variety of classifiers.

Approximately, 97.5% of the performance accuracy of the liver categorization is achieved with a 94.5% Continuous Interval (CI) of [0.6775 1.0000] and an error rate of 2.1%. The suggested method's performance is compared to that of two existing algorithms, and the sensitivity and specificity provide an overall average of 96% and 93%, respectively, with 95% Continuous Interval of [0.7513 1.0000] and [0.7126 1.0000] for the sensitivity and specificity

Figure 7 represents the performance metrics. When comparing the suggested technique to the current methods, the new method achieves superior results in terms of sensitivity, specificity, and accuracy. The accuracy of the classifier is used to estimate how successful it is by displaying the proportion of correct answers. Classifiers such as the ICNN and IANN perform much better in this situation than other classifiers. As a result, the ICNN classifier is capable of successfully classifying a greater amount of data than the other classifiers. The sensitivity and specificity of the classifier are used to evaluate its efficacy.

Figure 8 depicts the classification accuracy comparison results, with the proposed ICNN approach outperforming the other methods in terms of classification accuracy. The term “sensitivity” refers to how well a classification system performs regarding the number of adequately diagnosed benign tumors. In contrast, “specificity” refers to how well the classification system performs regarding the number of correctly classified malignant tumors. Compared to the other classifiers, the ICNN obtains a better level of sensitivity. Given that the goal of cancer detection is to determine whether a patient has cancer or not, which is indicated by the presence or absence of malignant tumors, the most fantastic accuracy and specificity are more significant in research. The rationale for this is that individuals diagnosed with cancer may be further studied to extend their lives, but those categorized as usual would stay unnoticed.

Figure 9 includes the ROC curves that are commonly used to evaluate the performance of binary classification algorithms, and they are also known as receiver operating characteristic curves. The performance of a classifier is represented graphically, rather than as a single numerical number, as is the case with most other metrics.

The computer vision field is built on the concepts of picture recognition and image generation. Despite the fact that both are developing domains, specific approaches from both subareas may sometimes create a dichotomy. Historically, the topic of deep learning (DL) was extensively popularized in discriminative image classification with the AlexNet architecture and picture synthesis with GANs and Variational Autoencoders, among other applications [34].

## 5. Conclusion and Future Work

Using abdominal CT medical images, a region-based image segmentation approach is provided to identify and segment the liver, which is the area of interest, as the region of interest. The suggested segmentation approach uses a local segmentation step, which provides an approximate boundary for the area of interest in the segmented region of interest. The level set approach fine-tunes this approximate border of the liver even further by using a region-based force function, which effectively stops the contours at weak or hazy margins. The algorithm's efficiency is measured using a variety of metrics and then compared to other conventional algorithms to see which is more efficient. Other soft computing approaches, such as image classification algorithms, may be investigated in the future to lower the computation processing time of liver tumor pictures. Testing against a variety of database pictures and multiple classifier models and optimization methodologies may help improve the accuracy of the liver tumor classification system. Other categorization parameters for liver tumor images are also being evaluated for inclusion in the classification process. Images of the same patient may be evaluated using a variety of imaging modalities, including ultrasound and 0.

To increase the accuracy of the classifier, hybrid classifier approaches may be used. It may be necessary for the liver tumor classification method to evaluate a more significant number of picture samples.

## Figures and Tables

**Figure 1:** Feature selection concerning liver image.

**Figure 2:** Flow of proposed work.

**Figure 3:** Feature Extraction using Dynamic Vector Warping (DVW).

**Figure 4:** Proposed improved convolutional neural network.

**Figure 5:** Partial Differential Technique with Input CT image of liver cancer cells.

**Figure 6:** Level Set Technique with Input CT image of liver cancer cells.

**Figure 7:** Performance metrics.

**Figure 8:** Confusion matrix obtained from training stage of input classifier.

**Figure 9:** ROC of input classifier.

**Table 1:** The feature values that were picked for 7 images.

Image	DVW	Local distance measure	Local cost measure	Entropy
1	858.000000	858.000000	858.000000	858.000000
2	84.000000	26.820513	0.040793	0.086247
3	32.000000	8.497948	0.197925	0.280892
4	25.000000	13.000000	0.000000	0.000000
5	13.000000	20.000000	0.000000	0.000000
6	8.497948	25.000000	0.000000	0.000000
7	26.820513	32.000000	0.000000	0.000000

**Table 2:** The classification results and performance with the existing classifiers.

Techniques	Accuracy	Sensitivity	Specificity	ROC
SVM	92.36	94.6	92.6	96.6
KNN	93.89	95.66	93.66	97.66
Naïve Bayes	94.36	95.98	96.98	98.98
CNN	95.6	95.36	97.36	97.36
ICNN	97.5	96	93	95

## Data Availability

The data that support the findings of this study are available on request from the corresponding author.

## Appendix

### A. Partial Differential Technique

  When the number of labels is zero, the following is true:
  S: labels 1 to N are used for markers, while labels *N* + 1 to NO are used for seed.
  Place a marker for each area labelled from 1 to N on the map.
  All pixels should be sorted in ascending order.
  For each pixel, begin by determining the number of labels that exist in N. (z)
  If the number of labelled pixels is zero, the current pixel obtains a new label, resulting in the creation of a new temporary area.
  Alternatively, Alternatively, if (labelled pixel = 1), the current pixel is assigned this label.
  Alternatively, Alternatively, if (labelled pixels ≥ 2), the current pixel is assigned an edge label.
  Alternatively, Alternatively, if (labelled pixels is a negative number)
  In order to merge the broken pictures and leaky images, the linear interpolation concept is used to interpolate them in order to locate the closest neighbor pixels. (It is also possible to wear a Mexican hat.)
  Else \s
  begin
  Combine all of the neighbors into a single area; the current pixel receives this name.
  End \s
  End

#### B. Level Set Methodology

  Initialize:
  Find the liver tumor cells interior blocks
  While (elements of *ϕ* is interchanged in the pixel values)
  For *i* = 1 to input number of speed iterations
  For each pixel *x* in *I*_*d*_(*A*)
  If (*d*_1_(*ϕ*) = = 1) switch x from *I*_*d*_(*A*) to *I*_*d*_(*A*′)
  Clean *I*_*d*_(*A*′)*at* *x*
  For *i* = 1 to output curvature selection
  For each pixel *x* in *I*_*d*_(*A*)
  If ((*ϕ*(*x*)) = = 1) switch *x* from *I*_*d*_(*A*′) to *I*_*d*_(*A*′)
  Clean *I*_*d*_(*A*′)*at* *x*
  End
  end
